The article "Exploring the Potential Mechanism of Xiaokui Jiedu Decoction for Ulcerative Colitis Based on Network Pharmacology and Molecular Docking" was retracted in 2023. Reasons: signs of a paper mill; compromised peer review; unreliable results or conclusions.

# Exploring the Potential Mechanism of Xiaokui Jiedu Decoction for Ulcerative Colitis Based on Network Pharmacology and Molecular Docking

**DOI:** 10.1155/2021/1536337

**Published:** 2021-10-25

**Authors:** Bin Wang, Yang Liu, Jianhui Sun, Nailin Zhang, Xiaojia Zheng, Qiquan Liu

**Affiliations:** Department of Spleen and Stomach Diseases, The First Affiliated Hospital of Hebei College of Traditional Chinese Medicine, Shijiazhuang, China

## Abstract

**Introduction:**

Network pharmacology is in line with the holistic characteristics of TCM and can be used to elucidate the complex network of interactions between disease-specific genes and compounds in TCM herbal medicines. Here, we investigate the pharmacological mechanism of Xiaokui Jiedu decoction (XJD) for the treatment of ulcerative colitis (UC).

**Methods:**

The Computational Systems Biology Laboratory Platform (TCMSP) database was searched and screened for the active ingredients of all drugs in XJD. The Uniport database was used to retrieve possible gene targets for the therapeutic effects of XJD. GeneCards, PharmGKB, TTD, and OMIM databases were used to retrieve XJD-related gene targets. A herb-compound-protein network and a protein-protein interaction (PPI) network were constructed, and hub genes were screened for Gene Ontology (GO) and Kyoto Encyclopedia of Genes and Genomes (KEGG) enrichment analyses. Finally, molecular docking was performed to validate the interrelationship between disease target proteins and active drug components.

**Results:**

A total of 135 XJD potential action targets, 5097 UC-related gene targets, and 103 XJD-UC intersection gene targets were screened. The hub gene targets of XJD that exert therapeutic effects on UC are *RB1*, *MAPK1*, *TP53*, *JUN*, *NR3C1*, *MAPK3*, and *ESR1*. GO enrichment analysis showed 741 biofunctional enrichments, and KEGG enrichment analysis showed 124 related pathway enrichments. Molecular docking showed that the active components of XJD (*β*-sitosterol, kaempferol, formononetin, quercetin, and luteolin) showed good binding activities to five of the six hub gene targets. *Discussion.* The active ingredients of XJD (*β*-sitosterol, kaempferol, formononetin, quercetin, and luteolin) may regulate the inflammatory and oxidative stress-related pathways of colon cells during the course of UC by binding to the hub gene targets. This may be a potential mechanism of XJD in the treatment of UC.

## 1. Introduction

Ulcerative colitis (UC) is a chronic nonspecific inflammatory disease of the rectum and colon of unknown etiology [1, 2]. The lesions mainly invade the mucosa and submucosa of the large intestine, with a continuous diffuse distribution, and the main clinical manifestations are diarrhea, mucopurulent stools, and abdominal pain.

In recent years, the incidence of ulcerative colitis (UC) has increased significantly, with 505 and 214 cases per 100,000 people in Europe and the United States, respectively, and the annual costs for UC-related screening and treatment amount to 12.5–29.1 billion euros and 8.1–14.9 billion dollars [3]. Aminosalicylic acid preparations, commonly used in the treatment of UC, exert anti-inflammatory effects mainly by affecting the metabolism of arachidonic acid and inhibiting prostaglandin synthesis, but their adverse effects are more frequent and their therapeutic effects are less satisfactory. Traditional Chinese medicine (TCM) has been shown to have potential advantages in UC treatment [1, 4, 5]. Hu et al. recently found that XJD was effective in treating UC by effectively regulating neuroendocrine factors, improving the intestinal immune response, and reducing patient symptoms [6]. However, the mechanisms involved in the field of UC treatment with XJD are still unknown.

Ulcerative colitis belongs to the category of “diarrhea” and “dysentery” in TCM and is mainly caused by damp-heat and a diet that damages the spleen and stomach. Network pharmacology is in line with the holistic characteristics of TCM and can elucidate the complex network of interactions between disease-specific genes and compounds in TCM herbal medicines [7–10].

In summary, our study combines network pharmacology, molecular docking, and cellular experimental analysis to investigate the pharmacological mechanism of XJD for UC treatment.

## 2. Methods

### 2.1. Screening for Active Ingredients and Potential Targets of XJD

In the Computational Systems Biology Laboratory Platform (TCMSP), herbs are searched separately (baitouweng (*Pulsatilliae radix*), huanglian (*Coptidis rhizoma*), huangbai (*Phellodendri chinensis cortex*), qinpi (*Fraxini cortex*), kusheng (*Sophorae flavescentis radix*), baiji (*Bletilla striata*), gegen (*Radix puerariae*), huaihua (*Sophora japonica* L.), xianhecao (*Agrimonia eupatoria*), and gancao (licorice)) [11]. The screening conditions are set as OB ≥ 30% and DL ≥ 0.18, and the active ingredients and related target information of the Chinese medicines were searched separately and screened based on pharmacokinetic absorption, distribution, metabolism, and excretion parameters. All potential targets were combined, and duplicates were excluded to obtain potential targets for the active ingredients of XJD.

### 2.2. XJD Active Ingredient Target Prediction

In the Uniport database (https://www.uniprot.org/), the Uniport KB function was used to search for human gene abbreviations related to the targets of the active ingredients of XJD and to obtain possible gene targets for the therapeutic effects of XJD.

### 2.3. UC-Related Disease Target Prediction

The GeneCards, OMIM, DrugBank, and PharmGKB databases were searched for relevant gene targets using the keyword “ulcerative colitis,” as shown in previous studies [4]. These potential XJD target genes were then linked to UC target genes to identify candidate targets.

### 2.4. Construction of the Herb-Compound-Protein Network and the Protein-Protein Interaction (PPI) Network

The R software package was used to plot the Venn diagram to obtain the intersection of drug and disease gene targets to achieve the likely therapeutic targets. These were then entered into the string system, and a protein-protein interaction (PPI) network was constructed with a confidence interval of ±0.950 [12]. Cytoscape was used for the herb-compound-protein network. Cytoscape's plugin CytoNCA calculated the parameters required to evaluate the functional importance of each node in the network [13]. This allowed further screening of the hub genes that were used to construct the PPI network. Next, the clusterProfiler package in R was used to perform Gene Ontology and KEGG pathway enrichment analyses on these hub genes (inclusion criteria: *p* value <0.05) [14, 15].

### 2.5. Molecular Docking

Molecular docking refers to the “docking theory” that relies on receptor-ligand interactions to predict the potential binding mode of a compound to a protein [16–18]. Hub genes in the PPI network were selected for molecular docking validation. We searched the PubChem database for 2D structures of possible active ingredients in XJD and the PDB database for 3D structures of the target proteins of the hub genes in the PPI network. The PyMOL software package was then used to remove water molecules and small molecule ligands from the target protein structures of the hub genes. AutoDockTools software was used to determine the active pockets at potential sites for molecular docking. Molecular docking was performed using AutoDock Vina software, and then PyMOL software was ultimately used to map and analyze the results of the lowest binding energy docking.

### 2.6. Animals and Drug Preparation

XJD is a combination of baitouweng (*Pulsatilliae radix*), huanglian (*Coptidis rhizoma*), huangbai (*Phellodendri chinensis cortex*), qinpi (*Fraxini cortex*), kusheng (*Sophorae flavescentis radix*), baiji (*Bletilla striata*), gegen (*Radix puerariae*), huaihua (*Sophora japonica* L.), xianhecao (*Agrimonia eupatoria*), and gancao (licorice). Animal welfare was carried out in strict accordance with the internationally accepted principles for laboratory animals (EEC Directive; 86/609/EEC). Sprague Dawley (SD) rats with a weight range of 270 ± 10 g were randomly divided into three groups according to body mass: blank group, XJD treatment group, and model group. Dosages administered were calculated with reference to the previous literature [19, 20]. The treatment group was given different doses of antidiarrhea pills by gavage, while the blank group and the model group were given an equal volume of saline by gavage twice a day for seven days. One hour after the last dose, blood was collected from the abdominal aorta under aseptic conditions. All animals were euthanised with thiopental sodium at the end of the experiment. The samples were placed in 10 mL centrifuge tubes, and the serum was inactivated in a 56°C water bath for 30 min, then filtered through a 0.22 *μ*m microporous membrane, and stored at −20°C for quantitative real-time PCR (qPCR). Followed by cDNA synthesis using the Prime-Script RT Master Mix (TaKaRa), total mRNA was isolated from the cell cultures using the Mini-BEST Universal RNA extraction kit (TaKaRa, Kyoto, Japan). And, qPCR assays were detected with PCR LightCycler480.

## 3. Results

### 3.1. XJD Active Ingredients and Potential Targets

The study flow chart is described in Figure 1. The preliminary search yielded 92 active ingredients of gancao (licorice), five active ingredients of xianhecao (*Agrimonia eupatoria*), six active ingredients of huaihua (*Sophora japonica* L.), four active ingredients of gegen (*Radix puerariae*), nine active ingredients of baiji (*Bletilla striata*), 45 active ingredients of kusheng (*Sophorae flavescentis radix*), three active ingredients of qinpi (*Fraxini cortex*), 27 active ingredients of huangbai (*Phellodendri chinensis cortex*), 11 active ingredients of huanglian (*Coptidis rhizoma*), and 12 active ingredients of baitouweng (*Pulsatilliae radix*). A total of 168 human gene targets corresponding to the active ingredients were searched through the Uniport database.

### 3.2. UC-Related Disease Target Prediction

Using the keyword “ulcerative colitis,” the GeneCards database retrieved 5,079 disease-related gene targets, the OMIM database retrieved 19 disease-related gene targets, the DrugBank database retrieved 13 disease-related gene targets, and the PharmGKB database retrieved 54 disease-related gene targets. A total of 5,097 UC-related gene targets were obtained by combining all disease-related gene targets (Figure 2(a)).

### 3.3. Construction of Herb-Compound-Protein Network and PPI Network

The Venn plot obtained the intersection of drug and disease gene targets and yielded 103 potential gene targets for XJD in the treatment of UC (Figure 2(b)). The herb-compound-protein network had 145 active ingredients associated with XJD for UC treatment, of which five with the highest number of corresponding gene targets included *β*-sitosterol, kaempferol, formononetin, quercetin, and luteolin (Figure 3). They were used to construct the PPI network of possible gene targets for XJD in the treatment of UC, as shown in Figure 4(a) (Figure S1). Figure 4(a) shows 78 nodes and 202 edges, Figure 4(b) shows 18 nodes and 72 edges, and Figure 4(c) shows seven nodes and 38 edges. The seven hub gene targets, *RB1*, *MAPK1*, *TP53*, *JUN*, *NR3C1*, *MAPK3*, and *ESR1*, were obtained after two analytical screens (Figures 4(b) and 4(c)).

### 3.4. Enrichment Analysis of Hub Genes

Gene screening and enrichment analysis of GO and KEGG were performed. Seven target genes were also analyzed for KEGG and GO enrichment, respectively, which is our focus. GO enrichment analysis showed that there were 741 biofunctional enrichments. GO functional enrichment analysis revealed that candidate target genes for UC were shown to be enriched in BPs (DNA-templated transcription, regulation of DNA-binding transcription factor activity, cellular response to starvation, cellular response to cadmium ion, response to starvation, regulation of telomerase activity, cellular response to nutrient levels, and cellular response to extracellular stimulus), CCs (nuclear chromatin, pseudopodium, nuclear/RNA polymerase II transcription factor complex, spindle, caveola, PML body, plasma membrane raft, and late endosome), and MFs (RNA polymerase II transcription factor binding, phosphoprotein binding, MAP kinase activity, phosphatase binding, disordered domain-specific binding, and phosphotyrosine residue binding) (*P* < 0.05; Figure 6(a)). KEGG enrichment showed that 124 related pathways were enriched. KEGG pathway analysis showed that those target genes were mainly involved in endocrine resistance, breast cancer, MAPK signaling pathway, hepatitis B, viral carcinogenesis, Kaposi's sarcoma-associated herpesvirus infection, melanoma, thyroid hormone signaling pathway, non-small-cell lung cancer, chemical carcinogenesis-receptor activation, pancreatic cancer, chronic myeloid leukemia, colorectal cancer, prostate cancer, neurotrophin signaling pathway, apoptosis, estrogen signaling pathway, thyroid cancer, gastric cancer, etc. (*P* < 0.05; Figure 6(b)). Six target genes (*ESR1*, *JUN*, *TP53*, *MAPK3*, *RB1*, and *MAPK1*) were enriched in the endocrine resistance pathway (Figure 6(a) and Figure S2), implying that they could be involved in the pathogenesis of UC.

### 3.5. Molecular Docking Analysis

Based on the above results, the active ingredients in XJD (*β*-sitosterol, kaempferol, formononetin, quercetin, and luteolin) were found to exhibit the same effects as *ESR1*, *JUN*, *NR3C1*, *MAPK1*, *MAPK3*, *RB1*, and *TP53* (Figure 7). These seven proteins were entered into the PDB database. For MOE molecular docking analysis, seven key target proteins (ESR1, JUN, NR3C1, MAPK1, MAPK3, RB1, and TP53) were selected (Figures 8(a)–8(e)) and were found to be related to *β*-sitosterol, kaempferol, formononetin, quercetin, and luteolin. Among them, *β*-sitosterol binds to *ESR1* with a binding energy of −5.8 kcal/mol, *JUN* at −5.4 kcal/mol, and *NR3C1* at − 4.3 kcal/mol. Kaempferol bound to *ESR1* with a binding energy of −7.1 kcal/mol and *JUN* at −5.5 kcal/mol. Formononetin bound to *ESR1* with a binding energy of −6.7 kcal/mol and to *JUN* at −5.7 kcal/mol. Quercetin bound to *ESR1* with a binding energy of −6.3 kcal/mol, *MAPK1* at −8.9 kcal/mol, *RB1* at −8.4 kcal/mol, and *TP53* at −8.3 kcal/mol. Luteolin bound to *ESR1* with a binding energy of −7.0 kcal/mol, *MAPK1* at −9.1 kcal/mol, *RB1* at −8.3 kcal/mol, and *TP53* at −8.3 kcal/mol (Table 1).

Molecular docking binding free energy less than −5.0 kcal/mol indicates strong binding activity, and that less than −7.0 kcal/mol indicates very strong binding activity. In the present study, 47% of targets (*n* = 8) had a molecular docking binding free energy less than −7.0 kcal/mol and 94% had less than −5 kcal/mol, indicating that the targets had good binding power with the components. Therefore, we suggest that XJD binds to these genes (*ESR1*, *JUN*, *NR3C1*, *MAPK1*, *MAPK3*, *RB1*, and *TP53*) very well and this may be the potential mechanism of XJD in the treatment of UC.

### 3.6. Effects of XJD Administration on the Expression Levels of FOS, TNF-*α*, and IL-1 mRNA in a UC Rat Model

FOS, TNF-*α*, and IL-1 are key proteins in the development of UC. RT-qPCR showed that the mRNA expression of FOS, TNF-*α*, and IL-1 was reduced in the XJD-treated group compared with the model group (*p* < 0.01) (Figure 9). The expression levels of FOS, TNF-*α*, and IL-1 mRNA in venous blood samples were significantly higher in the model group than in the blank group (*p* < 0.01). Therefore, the expression of key mRNAs (FOS, TNF-*α*, and IL-1) in UC was significantly downregulated after XJD administration. Our study reveals, to some extent, the pharmacological mechanism of XJD in the treatment of UC.

## 4. Discussion

Hu et al. recently found that XJD was effective in treating UC, with its ability to effectively regulate neuroendocrine factors, improve the intestinal immune response, and reduce patient symptoms [6]. Network pharmacology, animal experiments, and molecular docking approaches were used to systematically investigate the potential pharmacological mechanisms of XJD in UC treatment in this study.

A total of 135 potential action targets of XJD, 5,097 UC-related gene targets, and 103 XJD-UC intersection gene targets were screened, and 103 potential protein targets were found to be possible UC-related genes. The hub gene targets of XJD that exert therapeutic effects on UC are *RB1*, *MAPK1*, *TP53*, *JUN*, *NR3C1*, *MAPK3*, and *ESR1*. GO enrichment analysis showed 741 biofunctional enrichments, and KEGG enrichment analysis showed 124 related pathway enrichments. Molecular docking showed that the active components of XJD (*β*-sitosterol, kaempferol, formononetin, quercetin, and luteolin) showed good binding activity to six of the seven hub gene targets (*ESR1*, *JUN*, *NR3C1*, *MAPK1*, *RB1*, and *TP53*). *β*-Sitosterol, kaempferol, formononetin, quercetin, and luteolin have shown potential functions in the treatment of UC in many previous studies [21–25]. Variability and methylation patterns of *ESR1* were associated with the development of Crohn's disease in patients [1, 26]. The potential role of *JUN* and *MAPK1* [27, 28] and *NR3C1* [29] on UC is well known, and our study systematically revealed these links between them. Finally, the expression of key mRNAs (FOS, TNF-*α*, and IL-1) in UC was also significantly downregulated after XJD administration. Binding to these six genes, XJD therefore likely regulates the inflammatory response and pathways associated with the oxidative stress response in colon cells during the course of UC.

Many factors contribute to the development of UC, including genetic factors, environmental factors, bacterial infections, and hormonal drugs [30, 31]. Several studies have shown that intestinal barrier dysfunction and disruption of immune homeostasis within the intestinal mucosa are important causes of UC under pathological conditions [32, 33]. Under the pathological conditions of aggravated bacterial infection and UC, the tight junctions of intestinal epithelial cells are disrupted, cell permeability increases, and the intestinal barrier is destroyed, causing massive infiltration of immune cells and upregulation of inflammatory cytokine (i.e., TNF-*α*, IL-1, and FOS) expression, which promotes apoptosis of intestinal epithelial cells and increases permeability, further destroying the intestinal barrier and further aggravating local intestinal mucosal damage [30–33]. We found that the expression of inflammation-related factors (FOS, TNF-*α*, and IL-1) was downregulated after treatment of UC model mice with XJD. While our findings are quite valuable for UC treatment options, further experiments are still necessary to determine the specific mechanism of action of each active ingredient, and clinical studies need to be further refined.

## 5. Conclusions

In summary, XJD may have important therapeutic implications in treatment of UC lesions. It may be possible to correct colonic mucosal barrier dysregulation by regulating the expression of the core genes in UC.

## Figures and Tables

**Figure 1:** Abstract diagram of the research flow of this study.

**Figure 2:** (a) Venn diagrams of UC-related genes searched in the GeneCards, OMIM, DrugBank, and PharmGKB databases. (b) Venn diagram of drug target genes and UC-related target genes.

**Figure 3:** Herb-compound-protein network of UC and XJD.

**Figure 4:** PPI network and clustering of gene combinations at different levels (a–c).

**Figure 5:** (a) GO and (b) KEGG enrichment analysis of genes in Figure 4(b).

**Figure 6:** (a) GO and (b) KEGG enrichment analysis of genes in Figure 4(c).

**Figure 7:** Drug components-protein network diagram for potential mechanisms of XJD in the treatment of UC.

**Figure 8:** Schematic diagram of the docking of XJD active ingredients with NLRP3 target. *β*-Sitosterol (a), kaempferol (b), formononetin (c), quercetin (d), and luteolin (e).

**Figure 9:** Expression levels of FOS, TNF-*α*, and IL-1 mRNA of the rats. ^*∗∗*^/##*p* < 0.001.

**Table 1:** Virtual docking of five ingredients for UC targets.

Proteins	Binding energy (kcal/mol)				
	*β*-Sitosterol	Kaempferol	Formononetin	Quercetin	Luteolin
*ESR1*	−5.8	−7.1	−6.7	−6.3	−7.0
*JUN*	−5.4	−5.5	−5.7	−6.1	−5.6
*NR3C1*	−4.3	NA	NA	NA	NA
*MAPK1*	NA	NA	NA	−8.9	−9.1
*RB1*	NA	NA	NA	−8.4	−8.3
*TP53*	NA	NA	NA	−8.3	−7.9

## Data Availability

The data used to support this study are available from the corresponding author upon request.

## Supplementary Materials

Supplementary Materials Supplementary materials include Supplementary Figure 1 and Supplementary Figure 2. Figure S1: PPI network for XJD in the treatment of UC targets. Figure S2: (a) Endocrine resistance pathway and (b) MAPK signaling pathway.
